# Using Logistic Multivariate Analysis to Explore the Effects of Nursing and Psychological Factors on Motor and Cognitive Rehabilitation in Patients with Stroke: Based on a Retrospective Case-Control Study

**DOI:** 10.1155/2022/1411670

**Published:** 2022-08-19

**Authors:** Wenxin Lin, Liping Meng, Weimin Lou, Panpan Yang, Min Huang

**Affiliations:** Department of Rehabilitation Medicine, Zhejiang Hospital, Hangzhou 310000, China

## Abstract

**Objective:**

Based on a retrospective case-control study, logistic multivariate analysis was employed to explore the effects of nursing and psychological factors on the rehabilitation of motor and cognitive function in patients with stroke.

**Methods:**

A total of 200 stroke patients treated from February 2019 to April 2020 were enrolled in our hospital. According to the results of exercise and cognitive rehabilitation, the patients with good rehabilitation were divided into the control group (*n* = 140) and the research group (*n* = 60). The effects of nursing and psychological factors on the rehabilitation of motor and cognitive function in patients with stroke were analyzed.

**Results:**

First of all, we compared the general data. There were significant differences in terms of age, years of education, occupational status, payment methods of medical expenses, family income and the course of the disease, and the difference was statistically significant (*P* < 0.05). There was no significant difference in general data (*P* > 0.05). Secondly, we compared the nursing effective rates. The nursing effective rates of the study group were 10 cases, 15 cases, 12 cases, and 23 cases, and the nursing effective rate was 61.67%. In the control group, 78 cases were markedly effective, 33 cases were effective, 25 cases were general and 14 cases were ineffective, and the nursing effective rate was 90.00%. The effective rate of nursing in the study group was higher than that in the control group, and the difference was statistically significant (*P* < 0.05). There was no significant difference in anxiety and depression scores before nursing (*P* > 0.05), but they decreased after nursing. In addition, the scores of anxiety and depression in the study group were higher than those in the control group, and the difference was statistically significant (*P* < 0.05). There was no significant difference in motor function and cognitive function between prenursing and prenursing (*P* > 0.05); after nursing, the motor function increased and the score of cognitive function decreased. Furthermore, the motor function of the study group was lower compared to the control group, and the score of cognitive function of the study group was higher compared to the control group, and the difference was statistically significant (*P* < 0.05). The results of the Person correlation analysis showed that there was a significant correlation between nursing anxiety depression and the rehabilitation effect of motor cognitive function in stroke patients. The results of logistic regression analysis showed that age, family income, nursing efficiency, anxiety, and depression were the factors affecting the rehabilitation of motor and cognitive function in stroke patients.

**Conclusion:**

Age and family income may be the risk factors affecting the psychological mood of patients. Medical staff should pay attention to the negative emotion of patients and strengthen the nursing intervention of patients.

## 1. Introduction

Stroke, also known as cerebral apoplexy, is a sudden onset of symptoms lasting more than 24 hours or directly leading to death of local cerebrovascular blood circulation disorders [1]. Stroke, also known as stroke and cerebrovascular accident, is a group of diseases caused by sudden obstruction or rupture of cerebral vessels and brain tissue damage, including ischemic and hemorrhagic stroke [2]. Stroke is a common neurological disorder, which has become the second leading cause of death endangering human life in Europe. With the rapid development of the medical level, the survival rate of stroke patients has been remarkably promoted, but the subsequent high disability rate has become increasingly prominent. In accordance with the statistics of the World Health Organization, about 15 million patients worldwide suffer from stroke every year, about 5 million died after onset, and 5 million remain permanently disabled. In China, the annual incidence of stroke is about 250/100000, and the death rate is about 1.5 million. Its morbidity and mortality are among the highest in the world. In addition, 70%–80% of stroke survivors are unable to live independently because of disability [3]. The aging trend in China is becoming more and more serious. Due to the high-risk population of cerebrovascular disease in the elderly, the incidence of cerebrovascular disease remains high, which brings a huge burden to patients, patients' families, and society. For patients, the long-term illness will bring a variety of psychological problems, and these psychological problems will affect the physical recovery of patients.

Mental disorder is one of the most important secondary diseases of stroke [4]. The common psychological complications of stroke include depression, anxiety, mania, post-traumatic stress syndrome, emotional loss of control, apathy, and personality changes. The incidence of this kind of complication is high. In previous studies, the incidence of mental disorders caused by stroke varies greatly due to different psychological evaluation criteria, sampling locations, inclusion and exclusion criteria, and stroke course, ranging from 14.0% to 100% [5]. But overall, psychological problems are one of the important factors leading to a serious decline in the quality of life of patients with acute, convalescent, and chronic stroke. It has a significant impact on patients' functional recovery, disease development and complications, and even increases the risk of death [6]. The main manifestations of mental disorders caused by stroke are depression (PSD) and anxiety disorder (PSA). The fifth edition of the Diagnostic and Statistical Manual of Mental Disorders (DSM-5) defines depression as depression or lack of pleasure (loss of interest in things, unhappiness) lasting for more than two weeks and persistence of 4 or more of the following symptoms that affect normal daily life: sharp weight gain or sharp loss, insomnia or drowsiness, psychomotor agitation or deficiency, fatigue or lack of energy, sense of worthlessness or excessive guilt, lack of attention or loss of determination [7]. The incidence of depression is reported differently in related studies. The incidence of PSD is 25% to 65%. The risk of depression is the highest within 1 month after stroke, and some patients can recover on their own, but depressive symptoms persist in 1/3 of patients, especially in patients with severe depression, with an incidence of up to 30% in 1 year [7]. The meta-analysis indicated that the incidence of depression in patients with acute stroke was 28% (23% to 33%), 36% (29% to 43%) in recovery (2∼6 months), and 31% (26% to 37%) in chronic phase (more than half a year) [8]. The incidence of PSD is high, but it has not been paid enough attention to. Doctors usually pay attention to the improvement of patients' symptoms in the process of disease diagnosis, treatment, and rehabilitation, ignoring patients' psychological problems, resulting in delayed identification and treatment of PSD. Patients with depression can lead to a slow recovery of physical function, poor compliance for treatment and rehabilitation, increased medical consumption, reduced social activities, and reduced quality of life [9].

With the change of the concept of clinical nursing in China, the clinical nursing work with the core concept of “improving individual function and quality of life” pays more attention to the evaluation of physical and mental health of stroke patients, and has become an important link to enhance the rehabilitation effect of stroke patients [10]. The quality of life of stroke patients depends on the recovery of motor function and cognitive function. Rehabilitation training can effectively reduce the occurrence of stroke complications such as joint contracture, shoulder subluxation, shoulder-hand syndrome, and foot drop [11]. Stroke patients generally receive appropriate rehabilitation guidance and training during hospitalization or in professional rehabilitation institutions, and patients and caregivers can obtain certain rehabilitation knowledge, but due to the characteristics of stroke hemiplegia recovery, at least 45 minutes of moderate exercise rehabilitation training is carried out after discharge in order to ensure the rehabilitation effect during the rehabilitation period, it takes one day for patients who choose to rest at home. It is difficult to guarantee the quality of rehabilitation training. In addition, economic ability, traffic conditions, and other factors limit stroke patients to obtain timely professional rehabilitation guidance; patients are easy to miss the best opportunity for rehabilitation [10, 11]. Therefore, scholars have actively explored how to strengthen the functional recovery of stroke patients at home, although it has achieved certain results, it is still unable to meet the rehabilitation needs of patients. Based on this, this study focused on the effects of nursing and psychological factors on the rehabilitation of motor and cognitive function of stroke patients and carried out a logistic multivariate analysis to provide guidance for clinical stroke rehabilitation nursing.

## 2. Patients and Methods

### 2.1. General Information

A total of 200 stroke patients treated from February 2019 to April 2020 were enrolled in our hospital. According to the results of exercise and cognitive rehabilitation, the patients with good rehabilitation were divided into the control group (*n* = 140) and the research group (*n* = 60). With the permission of the Medical Ethics Association of our hospital, all patients signed the informed consent form.

Inclusion criteria were (1) in accordance with the diagnostic criteria revised by the 4th National Conference on Cerebrovascular Diseases in 1995 [12], the first stroke diagnosed by cranial CT and/or MRI examination; (2) 45–80 years old; (3) conscious (GCS >8), stable vital signs, no aphasia and the Montreal cognitive assessment (MoCA > 25); and (4) regular follow-up.

Exclusion criteria were (1) patients with a previous history of brain disease or injury; (2) patients with physical dysfunction before investigation; (3) patients with a previous history of mental illness, dementia, cognitive impairment, and severe organic diseases; (4) patients with blindness, deafness and mute; and (5) those who refused to participate in the follow-up survey after explanation.

### 2.2. Treatment Methods

#### 2.2.1. Nursing Methods

Rehabilitation nursing methods: rehabilitation training 30 minutes every time, twice a day, 5 days a week, regular training for 2 weeks, 10 minutes of active and passive training of shoulder joint, 10 minutes of active and passive training of elbow joint, and 10 minutes of wrist and hand function training. The convalesce should complete the traditional rehabilitation training on time and in accordance with the requirements of the experimental design and training.

#### 2.2.2. Psychological Factor

Selfrating anxiety scale is a psychological scale compiled by William W. K. Zung to analyze the degree of anxiety and its changes in the course of treatment [13]. After decades of repeated use and verification, the scale has become one of the most commonly used psychological measurement tools for psychological counselors and psychiatrists. It is mainly used to evaluate the curative effect, but not for diagnosis. The higher the score, the more serious the symptoms. The total score of anxiety is normal if the total score is less than 50, mild for 50, moderate for 61, and severe for more than 70. The number of negative items indicates how many items the subjects did not respond to, and the number of positive items indicates how many items the subjects responded to. Total rough score: the scores of 20 items are added together, and the demarcation is assigned to 40 points.

Selfrating Depression scale (SDS) is a selfrating scale consisting of 20 items and assigned into 4 grades. The prototype is the Depression scale compiled by W. K. Zung (1965). The cut-off value of the SDS standard score was 53, of which 53–62 was mild depression, 63–72 was moderate depression, and more than 73 was severe depression.

### 2.3. Observation Index

#### 2.3.1. General Information

Statistics of the two groups of patients' age, years of education, occupational status, medical expenses payment methods, family income, course of the disease, and gender.

#### 2.3.2. Motor Function Score

Using the functional Independence rating scale (FIM), which is proposed by the American Association of Rehabilitation Medicine and the Society of Physical Medicine and Rehabilitation. It is a scale widely adopted in the world to evaluate the ability of patients' daily activities. Including selfcare ability, sphincter control, transfer, action ability, communication, and social cognition five dimensions, a total of 18 items, the total score of 180.126, the higher the score, the better the functional independence of the patient. The FIM scale has good intragroup and intergroup reliability and good internal consistency.

#### 2.3.3. Cognitive Function Score

The patients were evaluated with the MoCA scale and the total score of MoCA was 30 points and the evaluation time was about 5–10 minutes. The score was higher than 25 considered normal. Cognitive impairment is considered below the standard score, which needs to be examined.

### 2.4. Statistical Analysis

The data of this study were processed by SPSS26.0 statistical software, the counting data were expressed by [*n* (%)], the chi-square test was used, the measurement data were expressed by mean ± standard deviation, *t*-test was used for comparison between groups, Pearson correlation analysis was used for normal distribution data, and Spearman correlation analysis was performed for skewness distribution data and grade data. Logistic regression was used to analyze the influencing factors. *P* < 0.05 indicated that the difference between groups is statistically significant.

## 3. Results

### 3.1. Comparison of General Data

First of all, compared with the general data there were significant differences in age years of education occupational status medical expenses payment mode family income and course of the disease, and the difference was statistically significant (*P* < 0.05). The gender difference was not significant and the data difference was not significant (*P* > 0.05). All the data results are indicated in Figure 1.

### 3.2. Comparison of Nursing Efficiency

Secondly, we compared the nursing effective rates. The nursing effective rates of the study group were 10 cases, 15 cases, 12 cases, and 23 cases, and the nursing effective rate was 61.67%. In the control group, 78 cases were markedly effective, 33 cases were effective, 25 cases were general and 14 cases were ineffective, and the nursing effective rate was 90.00%. The effective rate of nursing in the study group was higher than that in the control group, and the difference was statistically significant (*P* < 0.05). All the data results are indicated in Figure 2.

### 3.3. Comparison of Anxiety and Depression Scores

Thirdly, we compared the scores of anxiety and depression. Before nursing, there exhibited no significant difference (*P* > 0.05). The score for anxiety and depression in the study group was higher than that in the control group, and the difference was statistically significant (*P* < 0.05). All the data results are indicated in Table 1.

### 3.4. Comparison of Motor Function and Cognitive Function

Then, we compared the scores of motor function and cognitive function. Before nursing, there exhibited no significant difference (*P* > 0.05); After nursing, the motor function increased and the cognitive function score decreased. The score of motor function in the study group was lower than that in the control group, while the score of cognitive function in the study group was higher than that in the control group, and the difference was statistically significant (*P* < 0.05). All the data results are indicated in Table 2.

### 3.5. Correlation between Nursing and Psychological Factors and Rehabilitation Effect of Motor and Cognitive Function in Patients with Cerebral Apoplexy

Next, we analyzed the correlation between nursing and psychological factors and the rehabilitation effect on motor and cognitive function of stroke patients. The results of the Person correlation analysis showed that nursing anxiety and depression were significantly correlated with the rehabilitation effect of motor cognitive function in patients with stroke, and the difference was statistically significant (*P* < 0.05). All the data results are indicated in Table 3.

### 3.6. Logistic Regression Analysis of the Influencing Factors of Motor and Cognitive Rehabilitation in Patients with Cerebral Apoplexy

Finally, we conducted a logistic regression analysis on the influencing factors of motor and cognitive rehabilitation in stroke patients. The results of the logistic regression analysis indicated that age, family income, nursing efficiency, anxiety, and depression were the factors affecting motor and cognitive rehabilitation in stroke patients, and the difference was statistically significant (*P* < 0.05). All the data results are indicated in Table 4.

## 4. Discussion

Stroke is an obvious chronic and refractory disease, which seriously endangers human health and life. It is generally divided into embolic cerebral infarction, cerebral hemorrhage, subarachnoid hemorrhage, and other unclassified strokes [17]. According to the statistics updated by the American Heart Association (AHA) in 2013, the prevalence rate of stroke in the United States (2.8%), the incidence rate (790000/year), and the mortality rate (120000 in 2009) are still high [18]. Clinical manifestations are often transient or permanent brain dysfunction symptoms and signs, with high incidence, high disability rate, high recurrence rate, and high mortality rate. In 2011, AHA and the American Stroke Association (ASA) updated the Stroke Primary Prevention guidelines, indicating that stroke is the main cause of dysfunction, and 15∼30% of the survivors may be disabled [19]. In China, according to the guidelines for the Prevention and treatment of Cerebrovascular Diseases issued in 2007, it is estimated that there are about 2 million new stroke cases each year. About 75% of the survivors lost their ability to work and live to varying degrees, of which 40% were severely disabled [20]. In 2008, the third survey of the cause of death of residents in China indicated that cerebrovascular disease (mainly stroke) became the leading cause of death in the country. Therefore, the epidemiological situation of stroke in China is grim, and the responsibility for effective prevention and treatment of stroke is urgent and significant [21]. Rehabilitation training is the most effective way to enhance poststroke dysfunction in the treatment and rehabilitation of stroke. Meanwhile, it can strengthen the independence of life and the quality of life [22]. Stroke is a major event that threatens human physical and mental health. Stroke patients often start their own psychological defense mode to deal with psychological stress after the onset of stroke. Improper use of psychological defense will adversely affect the treatment and prognosis of stroke. Stroke psychological disorder is a curable complication, the use of antidepressants can partially promote the psychological symptoms of patients, but in addition to drug treatment, the study of the influencing factors of mental disorders after stroke can provide an important intervention direction for the prevention and control of such complications [23]. Therefore, scholars have actively explored how to strengthen the functional recovery of stroke patients at home, although it has achieved certain results, it is still unable to meet the rehabilitation needs of patients. Based on this, this study focused on the effects of nursing and psychological factors on the rehabilitation of motor and cognitive function of stroke patients and carried out a logistic multivariate analysis to provide guidance for clinical stroke rehabilitation nursing.

Anxiety disorder is a common psychological and mental symptom of patients after illness [24]. Usually, proper anxiety will promote patients' sense of selfprotection and enhance their healthy behavior. A certain degree of anxiety after a stroke is a normal psychological reaction of human beings after their lives are threatened. However, the high level of anxiety symptoms of psychological measurement will affect the quality of life of patients, bring more medical consumption, increase the risk of poor prognosis and family burden, and even be life-threatening in serious cases [24, 25]. The incidence of poststroke anxiety (PSA) was 8%∼29%, 20% in acute phase (13%∼26%), 23% in convalescent stage (19%∼27%), and 24% in chronic phase (19%∼29%) [26]. The main manifestations of PSA are excessive or irrational fear or worry, patients are often worried, upset, fidgeting, excessive vigilance, and often accompanied by autonomic nervous hyperactivity, such as palpitations, tremors, dizziness, sweating, and gastrointestinal discomfort. Some patients have panic attacks because the anxiety symptoms of some patients are similar to those of stroke and are ignored and the incidence of anxiety is reported less, the attention to anxiety symptoms is much lower compared to PSD. Studies indicate that 17% to 80% of PSA patients are also associated with PSD [26, 27]. So far, there are many studies on the influencing factors of PSA and depression. Scholars have investigated and verified the risk factors of psychological problems in stroke patients from different angles, but the results are still controversial [27]. The survey results of some scholars indicate that stroke patients generally have different types and degrees of psychological problems 2 weeks after illness (100%). This is related to the patient's education level, family background, stroke severity, and the degree of physical and speech disorders [28]. The investigation of other scholars indicated that the mood disorder after stroke was related to the type of stroke, the location of stroke focus, NIHSS score, and BI score at admission. However, some scholars believe that marital status, nerve injury, and daily activity ability have an influence on emotion [29]. There are also different research results on the effects of physical activity level and physical training on the psychology and spirit of stroke patients [30]. After the onset of stroke, the physique of stroke patients declined, and their cardiopulmonary endurance was about 50% of that of healthy people of the same age and sex, resulting in a serious lack of physical activity. The study on the psychological state of patients with stroke shows that rehabilitation exercise can improve the quality of life of patients, thus enhancing their psychological level [31]. However, there are also different research results. In a multicenter survey, we mainly observed the incidence, severity, and time process of anxiety and depression in stroke patients, and found that even if the patients' condition, characteristics, and exercise intensity were different. However, there exhibited no significant difference in the incidence and severity of anxiety and depression among patients in different rehabilitation centers, and patients with new psychological problems were found at each time. Some scholars have pointed out that some cognitive rehabilitation therapy can make patients' anxiety and depression states persist or even worsen, but the evidence intensity is not high and does not continue to demonstrate [31, 32].

Identifying patients' depressive symptoms and finding the risk of depression are very important for timely preventive measures, early and appropriate psychological intervention, and related treatment [32]. There are two explanations for the mechanism of poststroke depression PSD, one is physiological etiology, caused by brain lesions, and the other is psychogenic disorder, which is the patient's stress and emotional response to the disease. Therefore, the assessment of depression in stroke patients is different from other diseases because of the characteristics of neurological diseases. Mental and psychological diseases such as energy decline, fatigue, irritability, sleep disorders, and lack of attention in depression may also be neurological symptoms caused by brain diseases [32, 33]. Patients may have both neurological and psychosocial symptoms, which makes psychological assessment more difficult. Then, the functional impairment of patients, such as aphasia, anosognosia, confusion, or dementia, will affect the reliability of doctor-patient communication and patient reporting in the evaluation process, which also becomes an obstacle in the diagnosis of depression. Nursing and psychological factors are common research contents in the influencing factors of cognitive and motor rehabilitation of stroke, but there are a lot of controversies. Previous studies have indicated that stroke patients with poor cognitive and motor rehabilitation have a higher incidence of depression [33]. Clinical epidemiological investigation shows that there are differences in rehabilitation effect, nursing effective rate, and psychological factors among stroke patients, indicating that there are some differences in rehabilitation effect among stroke patients with different psychological states and nursing effects. After the onset of stroke, age and family income are also one of the factors affecting the mental state of patients. In addition, stroke often occurs in the middle-aged and elderly. Middle-aged and elderly women in menopause or postmenopause are more likely to induce psychological disorders due to the decrease in estrogen levels [33, 34]. Some studies have indicated that stroke is a risk factor for depression during the course of 3 years, which may be related to the individual's psychological defense mechanism during psychological stress [34]. In addition, regarding patients ≤ 50 years old and with good family income status, age ≤50 years old and with good family income status have better coping ability to deal with health problems [35]. Some scholars have also confirmed that the older the age is, the higher the risk of PSD is, especially within 2 months after onset, there is a significant correlation between age and depression [35, 36]. Although the incidence of stroke is younger, the physiological decline of the elderly makes the incidence of cerebrovascular diseases high in the elderly. The whole process of life development-transition theory holds that when an individual experiences transitional events in life, such as aging, sudden serious illness and other transitional events, personal role functions, goals, and life expectations will change due to the events. When the individual adjusts and adapts to the new life situation, there will be stress, the mild ones will only have emotional ups and downs, and the serious ones will develop into depression. Therefore, the inconsistency of the results in the study may come from the differences in the age of the subjects [36]. Further research should divide the age group reasonably and consider the impact of a variety of transitional events such as age, and good family income. The same idea can be found in the study put forward by other studies [37, 38]. They have applied new methods in the study, and the conclusions drawn can also give some support to this study. There are some limitations to this study. First, the sample size of this study is not large and it is a single-center study, so bias is inevitable. In future research, we will carry out multicenter, large-sample prospective studies, or more valuable conclusions can be drawn.

In summary, nursing and psychological factors have a certain influence on the rehabilitation of motor and cognitive function of stroke patients. There is a significant correlation between nursing effect and anxiety and depression in the rehabilitation of motor and cognitive function of stroke patients. Age and family income may be risk factors affecting patients' psychological emotions, suggesting that medical staff should pay attention to patients' negative emotions and strengthen nursing intervention for patients in order to promote the rehabilitation effect of motor and cognitive function in stroke.

## Figures and Tables

**Figure 1:** Comparison of general information of patients.

**Figure 2:** The effective rate of patient care in two groups.

**Table 1:** Comparison of anxiety and depression scores before and after nursing ($\bar{x}$ ± *s*, points).

Grouping	*N*	SAS		SDS	
		Before nursing	After nursing	Before nursing	After nursing
Control group	140	64.91 ± 4.12	41.39 ± 4.31	59.39 ± 3.12	45.31 ± 2.16
Research group	60	64.67 ± 4.12	54.91 ± 4.43	59.69 ± 3.42	54.49 ± 4.42
*t* value		0.377	20.160	0.605	19.725
*P* value		>0.05	<0.05	>0.05	<0.05

**Table 2:** Comparison of motor function and cognitive function scores before and after nursing ($\bar{x}$ ± *s*, points).

Group	*N*	Motor function		Cognitive function	
		Before nursing	After nursing	Before nursing	After nursing
Control group	140	44.69 ± 4.42	83.96 ± 14.12	25.24 ± 2.12	15.67 ± 1.66
Research group	60	44.91 ± 4.33	68.93 ± 10.31	25.21 ± 2.41	20.49 ± 1.22
*t* value		0.324	7.434	0.087	20.256
*P* value		>0.05	<0.05	>0.05	<0.05

**Table 3:** Correlation between nursing and psychological factors and rehabilitation effect of motor and cognitive function in patients with cerebral apoplexy.

Factors	*r*	*P*
Nursing	0.881	<0.05
Anxiety	−0.685	<0.05
Depression	−0.866	<0.05

**Table 4:** Logistic regression analysis of the influencing factors of motor and cognitive rehabilitation in patients with cerebral apoplexy.

Factors	*b*	S.E	Chi-square value	*P*	OR	95% CI for OR
Age	2.122	0.553	14.724	0.000	8.348	2.824–24.677
The number of years of education	1.221	1.432	0.727	0.394	3.391	0.205–56.133
Occupational condition	1.244	1.221	1.038	0.308	3.469	0.317–37.984
Payment method of medical expenses	2.561	1.874	1.868	0.172	12.949	0.329–509.811
Household income status	2.141	0.532	6.622	0.000	12.807	4.514–36.333
Nursing effective rate	2.550	0.532	22.975	0.000	12.807	4.514–36.333
Anxiety	−2.313	0.422	30.042	0.000	0.099	0.043–0.226
Depression	−2.144	0.451	22.599	0.000	0.117	0.048–0.284

## Data Availability

The datasets used and analyzed during the current study are available from the corresponding author upon reasonable request.

## References

[1] Zhang Y., Xie J., Wang L. (2021). Effect of improved food intake training based on dietary preference on swallowing function in patients with stroke. *Chinese Journal of physical Medicine and Rehabilitation*.

[2] Zhang Y., Li Y., Huang Z. (2021). Effect of continuous nursing of regional medical association on self-nursing ability and quality of life of stroke patients. *Journal of Nursing*.

[3] Huang C., Liu D., Zhu J. (2021). Observation on the effect of intervention based on multidisciplinary collaborative diagnosis and treatment in patients with acute ischemic stroke. *Nursing Journal*.

[4] Zheng J., Hu H., Li D. (2021). Observation and nursing care of patients with acute macrovascular occlusive ischemic stroke after thoracoscopic lobectomy. *PLA Journal of Nursing*.

[5] Ge L., Fang Y., Rao S. (2022). A retrospective case-control study on late failure of arteriovenous fistula in hemodialysis patients and prediction of risk factors. *Computational and Mathematical Methods in Medicine*.

[6] Maggio M. G., Latella D., Maresca G. (2019). Virtual reality and cognitive rehabilitation in people with stroke: An overview. *Journal of Neuroscience Nursing*.

[7] Loetscher T., Potter K. J., Wong D., das Nair R. (2019). Cognitive rehabilitation for attention deficits following stroke. *Cochrane Database System Review*.

[8] Sarfo F. S., Ulasavets U., Opare-Sem O. K., Ovbiagele B. (2018). Tele-rehabilitation after stroke: an updated systematic review of the literature. *Journal of Stroke and Cerebrovascular Diseases*.

[9] Renton T., Tibbles A., Topolovec-Vranic J. (2017). Neurofeedback as a form of cognitive rehabilitation therapy following stroke: A systematic review. *PLoS One*.

[10] Wu Q., Zhou J., Wang S. (2021). Mediating effect of rehabilitation self-efficacy between PSD and post-stroke fatigue in elderly stroke convalescent patients. *Nursing Journal*.

[11] Kim Sun Ho (2021). Effects of dual transcranial direct current stimulation and modified constraint-induced movement therapy to improve upper-limb function after stroke: a double-blinded, pilot randomized controlled trial. *Journal of Stroke and Cerebrovascular Diseases*.

[12] Xue X. (2021). Application of hemiplegic limb rehabilitation training in nursing care of patients with cerebral infarction and its effect on quality of life-- comment on Clinical Nursing of Neurology. *Clinical Pharmacology and Therapeutics in China*.

[13] Kanika K., Singh G. (2021). Commentary on: effect of a comprehensive E-rehabilitation Intervention alongside conventional stroke rehabilitation on disability and Health-Related quality of life: a Pre-Post comparison. *Journal of Rehabilitation Medicine*.

[14] Matsushita T., Nishioka S., Taguchi S. (2021). Effect of improvement in sarcopenia on functional and discharge outcomes in stroke rehabilitation patients. *Nutrients*.

[15] Thornton M., Jennifer H., Krista B., Dyks T., Finestone H., MacKay-Lyons M. (2021). Development of a digital learning program for physiotherapists to enhance clinical implementation of aerobic exercise in stroke rehabilitation. *Archives of Physiotherapy*.

[16] Tay M. (2021). Hospital readmission in stroke survivors one year versus three years after discharge from inpatient rehabilitation: prevalence and associations in an asian cohort. *Journal of Rehabilitation Medicine*.

[17] Low Michelle A., Power E., Margaret McG. (2021). Sexuality after stroke: exploring knowledge, attitudes, comfort and behaviours of rehabilitation professionals. *Annals of physical and rehabilitation medicine*.

[18] Raff C., Mary C., Chris C., Lamont R., Dean S., Tarrant M. (2021). Challenges of recruiting patients into group-based stroke rehabilitation research: reflections on clinician equipoise within the singing for people with aphasia (SPA) pilot trial. *Frontiers in Psychology*.

[19] Song R., Park M., Jang T., Oh J., Sohn M. K. (2021). Effects of a tai chi-based stroke rehabilitation program on symptom clusters, physical and cognitive functions, and quality of life: a randomized feasibility study. *International Journal of Environmental Research and Public Health*.

[20] Calabrò R. S., Sorrentino G., Cassio A. (2021). Robotic-assisted gait rehabilitation following stroke: a systematic review of current guidelines and practical clinical recommendations. *European Journal of Physical and Rehabilitation Medicine*.

[21] Lim J., Lim T., Lee J., SimChangYoonJung H. (2021). Patient-specific functional electrical stimulation strategy based on muscle synergy and walking posture analysis for gait rehabilitation of stroke patients. *Journal of International Medical Research*.

[22] Ahmad Ainuddin H., Romli M. H., Hamid T. A., S F Salim M., Mackenzie L. (2021). An exploratory qualitative study with older Malaysian stroke survivors, caregivers, and healthcare practitioners about falls and rehabilitation for falls after stroke. *Frontiers in Public Health*.

[23] van MeijerenPont W., Tamminga Sietske J., Goossens Paulien H. (2021). Societal burden of stroke rehabilitation: costs and health outcomes after admission to stroke rehabilitation. *Journal of Rehabilitation Medicine*.

[24] Norouzi Gheidari N., Archambault Philippe S., Monte Silva K. (2021). Feasibility and preliminary efficacy of a combined virtual reality, robotics and electrical stimulation intervention in upper extremity stroke rehabilitation. *Journal of Neuroengineering and Rehabilitation*.

[25] Bahia H., Anita P., Chiara C. (2021). Predictors of function, activity, and participation of stroke patients undergoing intensive rehabilitation: a multicenter prospective observational study protocol. *Frontiers in Neurology*.

[26] Lee D., Bae Y. (2021). Short-term effect of kinesio taping of lower-leg proprioceptive neuromuscular facilitation pattern on gait parameter and dynamic balance in chronic stroke with foot drop. *Healthcare*.

[27] Breen Joan C. (2021). Abstract P209: community-based outpatient stroke rehabilitation program achieves excellent return to work outcomes: characteristics and rehabilitation outcomes of stroke survivors who return to work. *Stroke*.

[28] Annie R., Ariane D., Morissette Gravel Anne S. (2021). Inclusion of relatives in stroke rehabilitation: perception of quality of services they received in the context of early supported discharged (ESD), in- and out-patient services. *Topics in Stroke Rehabilitation*.

[29] Hara T., Aturan S., McIntyre A., Burhan A. M. (2021). The effect of non-invasive brain stimulation (NIBS) on attention and memory function in stroke rehabilitation patients: a systematic review and meta-analysis. *Diagnostics*.

[30] Jeffares I., Merriman N. A., Doyle F., HorganHickey A. (2021). Inclusion of stroke patients in expanded cardiac rehabilitation services: a cross-national qualitative study with cardiac and stroke rehabilitation professionals. *Disability & Rehabilitation*.

[31] Kumar A., Fang Q., Elena P. (2021). The influence of psychological and cognitive states on error-related negativity evoked during post-stroke rehabilitation movements[J]. *BioMedical Engineering Online*.

[32] Edwards Jodi D., Black Sandra E., Shaun B. (2021). Canadian platform for trials in noninvasive brain stimulation (CanStim) consensus recommendations for repetitive transcranial magnetic stimulation in upper extremity motor stroke rehabilitation trials. *Neurorehabilitation and Neural Repair*.

[33] van Bloemendaal M., Bus S. A., Nollet F., Geurts A. C., Beelen A. (2021). Feasibility and preliminary efficacy of gait training assisted by multichannel functional electrical stimulation in early stroke rehabilitation: a pilot randomized controlled trial. *Neurorehabilitation and Neural Repair*.

[34] Cai H., Lin T., Chen L., Weng Zhu ChenCai G. (2021). Evaluating the effect of immersive virtual reality technology on gait rehabilitation in stroke patients: a study protocol for a randomized controlled trial. *Trials*.

[35] Wolf Timothy J. (2021). Doherty Meghan, Boone Anna, et al. Cognitive oriented strategy training augmented rehabilitation (COSTAR) for ischemic stroke: a pilot exploratory randomized controlled study. *Disability and Rehabilitation*.

[36] Kevdzija M., Marquardt G. (2021). Stroke patients’ nonscheduled activity during inpatient rehabilitation and its relationship with the architectural layout: a multicenter shadowing study. *Topics in Stroke Rehabilitation*.

[37] Javeed A., Sanam Shahla R., Zhou S., Riaz R., Khan S. U., Kwon S. J. (2020). Heart risk failure prediction using a novel feature selection method for feature refinement and neural network for classification. *Mobile Information Systems*.

[38] Zhao Z., Feng L. (2022). Logistic regression analysis of risk factors and improvement of clinical treatment of traumatic arthritis after total hip arthroplasty (THA) in the treatment of acetabular fractures. *Computational and Mathematical Methods in Medicine*.

